This article has been retracted.

# MicroRNA-let-7 Targets HMGA2 to Regulate the Proliferation, Migration, and Invasion of Colon Cancer Cell HCT116

**DOI:** 10.1155/2021/2134942

**Published:** 2021-09-15

**Authors:** Zheng Chen, Jiheng Liu

**Affiliations:** ^1^Department of General Surgery, The First Hospital of Changsha, Changsha, Hunan 410005, China; ^2^Department of Hematology & Oncology, The First Hospital of Changsha, Changsha, Hunan 410005, China

## Abstract

**Objective:**

To investigate the effect of microRNA-let-7 (miR-let-7) on the proliferation, migration, and invasion of colon cancer cell HCT116 in vitro and its regulatory mechanism on downstream HMGA2.

**Methods:**

It was planned to synthesize miR-let-7 overexpression (mimics) and interference expression (inhibitor) and transiently transfect colon cancer cell HCT116, detect the expression levels of miR-let-7 and HMGA2 in the cells after transfection and the targeted regulation effect of miR-let-7 on HMGA2, then detect the effect of upregulation/downregulation of miR-let-7 on HMGA2, and detect the proliferation, migration, and invasion of HCT116 cells.

**Results:**

The expression of miR-let-7 was downregulated, and the expression of HMGA2 was upregulated in HCT116. The expression of miR-let-7 increased significantly after HCT116 was transfected with miR-let-7 mimics. The expression of miR-let-7 decreased significantly after HCT116 was transfected with miR-let-7 inhibitor. The bioinformatics websites predicted that miR-let-7 has a binding site with HMGA2, and the dual-luciferase reporter gene experiment detected that miR-let-7 has a targeting relationship with HMGA2. The expression of HMGA2 decreased after HCT116 was transfected with miR-let-7 mimics; the expression of HMGA2 increased after HCT116 was transfected with miR-let-7 inhibitor. After upregulating miR-let-7, the proliferation, migration, and invasion ability of HCT116 was weakened. After miR-let-7 was inhibited, the proliferation, migration, and invasion ability of HCT116 was enhanced.

**Conclusion:**

Abnormal expression of miR-let-7 is an important factor affecting the proliferation, migration, and invasion of HCT116 cells, and it can promote or inhibit the biological behavior of cancer cells by targeting the expression of HMGA2. This study provides ideas for the drug development of new gene targets.

## 1. Introduction

The morbidity and mortality of colon cancer are, respectively, the 3rd and 4th among systemic malignant tumors. With the changes in people's eating habits and structure and the aging of the population, the morbidity and mortality are on the rise [1, 2]. The clinical treatment plan for colon cancer is mainly a comprehensive treatment of surgical resection combined with radiotherapy and chemotherapy. Because of the lack of specific manifestations of colon cancer in the early stage, most patients are already in the middle and advanced stages at the time of diagnosis. Recurrence and metastasis are the main factors affecting the efficacy [3]. Looking for new treatment methods and strategies to improve the treatment effect of colon cancer has become a hot spot in clinical research.

Gene therapy is a new concept of cancer treatment, and clarifying the biological genetic characteristics that affect the incidence and progression of colon cancer can provide new evidence for gene therapy and prognosis improvement. The occurrence of colorectal cancer is related to the abnormal expression of multiple genes. Regulating the expression of certain key genes during tumorigenesis to block malignant transformation is one of the effective means to control tumors [4]. Recent research evidence shows that high mobility group protein A2 (high mobility group AThook2, HMGA2) is upregulated in a series of epithelial malignant tumors. As its expression level increases, it significantly affects the prognosis of patients with malignant tumors [5]. Further tumor molecular biology studies have shown that HMGA2 has a regulatory role in the progression of tumors, such as cell proliferation and cycle adjustment, epithelial-mesenchymal transition, and maintenance of tumor stem cell function. It has played an important role and may become a new specific diagnostic marker and target of antitumor drug therapy [6]. Studies have shown that there is overexpression of HMGA2 in colon cancer tissues, and it is related to the clinical characteristics and prognosis of patients [7]. Therefore, HMGA2 is considered to be a potentially important tumor marker of colon cancer.

miRNA participates in the regulation of a series of cellular events including cell proliferation, development, cell metabolism, and apoptosis. Therefore, the dysfunction of miRNA will lead to the occurrence and development of malignant tumors [8, 9]. MicroRNA-let-7 (miR-let-7) is considered to be a tumor suppressor. Studies have shown that miR-let-7 is underexpressed in tumors, including colon cancer, and is closely related to the development of tumors [10–12]. Therefore, we speculate that the biological role of colon cancer may be related to the regulation of miR-let-7. Therefore, the role of miR-let-7 in colon cancer and whether it participates in the regulation of HMGA2 is worthy of in-depth study, providing a potential molecular target for gene therapy of colon cancer. In this study, artificial chemically synthesized miR-let-7 mimics and inhibitors were transfected into colon cancer HCT116 cells to explore the regulation of miR-let-7 on HMGA2 and its effect on colon cancer HCT116 cell proliferation, invasion, and apoptosis. We report the results as follows.

## 2. Materials and Methods

### 2.1. Cells and Materials

Human normal epithelial cell FHC and human colon cancer cell line HCT116 were purchased from Research Domain Biotechnology (Shanghai) Co., Ltd.; HMGA2 antibody was purchased from Abcam, USA; Matrigel glue was purchased from Sigma; Transwell chamber was purchased from Corning, USA; standard protein, electrochemical electrochemiluminescence (ECL) reaction detection kit and MTT kit were purchased from Shanghai Biyuntian Biotechnology Co., Ltd.; fetal bovine serum (FBS) DMEM medium was purchased from Gibco, the United States; Lipofectamine 2000 transfection reagent was purchased from the United States Invitrogen; Trizol and reverse-transcription kits were purchased from Wuhan Kehaojia Biotechnology Co., Ltd.; and RT-PCR kits were purchased from Takara, Japan.

### 2.2. Cell Culture

HCT116 cells were grown adherently in DMEM medium containing 10% FBS penicillin (100 *μ*g/ml) and streptomycin (100 *μ*g/ml) and subcultured in an incubator with 37°C 5% CO_2_ and saturated humidity.

### 2.3. Cell Transfection and Grouping

We took HCT116 cells in logarithmic growth phase, trypsinized and centrifuged at 1000*g* for 2 minutes, collected the cells, adjusted the cell density to 1 × 10^5^/well, and inoculated them into a 6-well cell culture plate. Each well was added with 2 ml cell suspension and cultured for 24 h under 37°C and 5% CO_2_ conditions. The cells were divided into 4 groups, namely, blank control group without transfection, mimic-NC group transfected with miR-let-7 mimic negative control, miR-let-7-mimic group transfected with miR-let-7 mimic, inhibitor-NC group transfected with miR-let-7 inhibitor negative control, and miR-let-7-inhibitor group transfected with miR-let-7 inhibitor; the transfection process was carried out according to Lipofectamine 2000 instructions.

### 2.4. qRT-PCR Detected the Expression Levels of miR-let-7 and HMGA2 mRNA in Cells

The cell sample was taken out, and the 6-well plate was used to inoculate the density of 2 × 10^5^ cells/well. The total RNA was extracted from the cells by the TRIzol method, and the reverse-transcription kit was used to reverse-transcribe cDNA from the above RNA, and finally miR-let-7 and other primers were used. Real-time qPCR was performed on the real-time PCR system. 2 *μ*l of the reverse-transcription product was taken out as a PCR reaction template, and the content of miR-let-7 was detected by fluorescence quantitative method. The reaction conditions were 95 denaturation for 10 s, 58 annealing for 10 s, 72 extension for 10 s, and the number of cycles set to 40. The primer sequences are shown in Table 1. The 2^-△△Ct^ method was used to analyze the quantitative results. △Ct (*n*) = Ct target gene (*n*)-Ct internal reference gene (*n*), △△CT (*n*) = △Ct (*n*)-△Ct (1).

### 2.5. Western Blot Detected the Expression Level of HMGA2 Protein

The total protein of each group of cells was extracted, the protein concentration was determined by the standard curve method, and sodium dodecyl sulfate-polyacrylamide gel electrophoresis (SDS-PAGE) was performed. After transfer, the membrane was blocked with 5% skim milk at room temperature for 1 hour, and the primary antibody was added. The primary antibody (HMGA2, 1 : 500, GAPDH: 1 : 1000) was discarded overnight at 4 degrees Celsius, and the nitrocellulose membrane was washed 3 times with Tris buffered saline (TBS) (high salt) for 10 minutes each time; then the secondary antibody was added, and the second antibody was used at room temperature for 2 hours. After the resistance, the NC membrane was cleaned 3 times with TBS, each time for 10 minutes. The exposure processing was performed according to the ECL instructions and the QuantityOne software was used for grayscale analysis. The relative expression of HMGA2 protein was expressed as the ratio of the gray value of HMGA2 to the gray value of the same group of GAPDH.

### 2.6. MTT Detected the Proliferation Activity of HCT116 Cells

48 h after transfection, the HCT116 cell suspension prepared by trypsinization method was transferred to a 96-well plate, and the cell density was adjusted. Each well contained 1 × 10^4^ cells, and each group had 6 multiple wells. 24 h, 48 h, and 72 h after inoculation, 20 *μ*l of MTT was added to each well; after 4 h of culturing, the supernatant was discarded, and 100 *μ*l of DMSO was added to dissolve the precipitate for 15 min, and the color was compared with the microplate reader. The absorbance value at 490 nm was recorded.

### 2.7. Wound Healing Test Detected the Migration of HCT116 Cells

The colon cancer cells in the logarithmic growth phase of each group were inoculated into a 6-well plate, and a 200 *μ*L yellow pipette tip was used in the middle of the 6-well plate to draw a wound through the culture hole. The wounds of each hole needed to be kept consistent, the culture medium was discarded, and the PBS was rinsed 3 times. After culturing for 48 hours, the suspended cells were discarded, and the wells were photographed to observe the cell migration near the wound. Judge the migration ability of cells based on the distance of the wound.

### 2.8. Transwell Method Detected the Invasion of HCT116 Cells

After transfection, 1 × 10^5^ HCT116 cells were taken out and seeded in the Transwell plate chamber, 160 *μ*l per well, 40 *μ*l 20% ASPS serum was added, and diluted Matrigel (3.9 *μ*g/*μ*l) 60–80 *μ*l was added to the polycarbonate membrane in the upper chamber, set 37°C 30 min to polymerize Matrigel into a gel. 800 *μ*l RMPI1640 medium was added to the lower chamber and cultured for 24 h. The number of cells in the subbasement membrane compartment was counted, and the number of cells passing through the basement membrane in a field of view was randomly selected under a 400 microscope, and the average was taken.

### 2.9. Statistical Methods

SPSS23.0 software was used for statistical analysis, and GraphPad Prism 8 was used for statistical mapping. The measurement data were expressed as mean ± standard deviation, the comparison between groups was performed by Student's *t*-test, and the one-way analysis of variance was used for comparison. *P* < 0.05 indicates that the difference is statistically significant.

## 3. Results

### 3.1. The Expression of miR-let-7 and HMGA2 in Colon Cancer Cell HCT116

The results showed that, compared with FHC cells, the expression of miR-let-7 mRNA in colon cancer cell HCT116 was reduced, and the expression of HMGA2 mRNA and protein was increased (*P* < 0.05, Figures 1(a)–1(c)) It is suggested that the expression of miR-let-7 is downregulated and the expression of HMGA2 is upregulated in colon cancer cell HCT116.

### 3.2. The Expression of miR-let-7 in Colon Cancer Cell HCT116 after Transfection

The results found that, compared with the blank control group, the expression of miR-let-7 mRNA in the mimic-NC group and the inhibitor-NC group had no significant change (*P* > 0.05). Compared with the mimic-NC group, the expression level of miR-let-7-mimic miR-let-7 mRNA was significantly higher; compared with the inhibitor-NC group, the expression level of miR-let-7-inhibitor miR-let-7 mRNA was significantly reduced (*P* < 0.05, Figures 2(a) and 2(b)). This suggests that colon cancer cell HCT116 successfully upregulates and inhibits miR-let-7 vector after transfection.

### 3.3. miR-Let-7 Had a Targeting Relationship with HMGA2

The results of the dual-luciferase report showed that the luciferase activity of WT-HMGA2 transfected with miR-let-7-mimic decreased, and the luciferase activity of WT-HMGA2 transfected with miR-let-7-inhibitor increased (*P* < 0.05), while MUT-HMGA2 did not change significantly (*P* > 0.05, Figure 3). This suggests that miR-let-7 has a targeting relationship with HMGA2.

### 3.4. The Regulatory Effect of miR-let-7 on HMGA2

The above experiments had proved that miR-let-7 has a targeting relationship with HMGA2. In order to verify this result, we used qRT-PCR to detect the upregulation and suppression of HMGA2 mRNA and protein expression levels after cell transfection with miR-let-7 vector. The results showed that, compared with the blank control group, the expression of HMGA2 mRNA in the mimic-NC group and the inhibitor-NC group did not change significantly (*P* > 0.05); compared with the mimic-NC group, the expression of miR-let-7-mimic HMGA2 mRNA and protein expression level was significantly reduced; compared with the inhibitor-NC group, the miR-let-7-inhibitor HMGA2 mRNA and protein expression level was significantly increased (*P* < 0.05, Figures 4(a)–4(d)). It is suggested that miR-let-7 can target the expression of HMGA2.

### 3.5. The Effect of Upregulation of miR-let-7 on the Proliferation, Migration, and Invasion of Colon Cancer Cell HCT116

The results showed that, compared with the blank control group, the mimic-NC group had no significant changes in cell proliferation, migration, and invasion abilities (*P* > 0.05). Compared with the mimic-NC group, the miR-let-7-mimic group had weaker cell proliferation, migration, and invasion abilities (*P* < 0.05, Figures 5(a)–5(c)). It is suggested that upregulation of miR-let-7 can inhibit the biological behavior of colon cancer cell HCT116.

### 3.6. The Effect of Inhibiting miR-let-7 on the Proliferation, Migration, and Invasion of Colon Cancer Cell HCT116

The results showed that, compared with the blank control group, the inhibitor-NC group had no significant changes in cell proliferation, migration, and invasion abilities (*P* > 0.05). Compared with the inhibitor-NC group, the miR-let-7-inhibitor group had enhanced cell proliferation, migration, and invasion abilities (*P* < 0.05, Figures 6(a)–6(c)). It is suggested that inhibition of miR-let-7 can promote the proliferation, migration, and invasion of colon cancer cell HCT116.

## 4. Discussion

Among the global malignant tumors, the incidence rate of colon cancer has risen to the third place, and the mortality rate ranks the first. The incidence of patients is mainly concentrated in the 40–50-year-olds [13, 14]. The occurrence of colon cancer involves multiple stages such as multiple protooncogenes and tumor suppressor genes and is the result of the interaction of multiple oncogenes. When the balance between protooncogene and tumor suppressor gene is broken, the protooncogene is overexpressed, the tumor suppressor gene loses its activity, and the immune mechanism cannot control the development of cancer cells and cancer is formed [15]. miRNAs can directly target mRNAs to regulate gene expression, leading to translational inhibition or instability [16].

miRNA (microRNA) is an endogenous noncoding small RNA with a length of approximately 22 nucleotides. miRNA can recognize and bind to the sequence of the 3′-untranslated region of the target gene and inhibit the target gene by inhibiting translation and inducing mRNA degradation [17]. Although only more than 700 miRNAs have been found in the human genome so far, since each miRNA can regulate hundreds of target genes, miRNAs can regulate more than 30% of human genes. miRNAs can promote the growth, proliferation, metastasis, and invasion of tumors and play the role of tumor growth factors. Researchers call this kind of tumor-inducing miRNAs cancer-promoting genes, whereas the miRNAs that exert tumor-inhibiting effects are called tumor suppressor genes [18, 19]. Studies have shown that miR-let-7 inhibits the occurrence of a variety of cancers, such as breast cancer [20], bladder cancer [21], and colon cancer [22]. However, the specific mechanism by which miR-let-7 miRNA regulates the progression of colon cancer has not yet been fully elucidated.

In order to further study the downstream regulatory mechanism of oncogene miR-let-7 and its role in tumors, we analyzed the 3 untranslated regions of miR-let-7 gene mRNA through bioinformatics software and found a potential binding of HMGA2 site. HMGA2 is a structural transcription factor. It does not have the ability to regulate transcription, but it can combine with the enriched region on the regulated gene DNA through its own unique structure or directly participate in the action of certain transcription factors, by changing these transcriptions. The DNA conformation of the factor enhances or inhibits its transcriptional activity. Studies have shown that HMGA2 plays an important role in physiological processes such as embryonic developmental cell proliferation, diabetes, obesity, and height regulation and is also closely related to the occurrence and development of tumors [23–25]. Studies have shown that the let-7a/HMGA2 axis plays a key role in regulating the migration and invasion of tongue squamous cell carcinoma, which may lay the foundation for the relationship between let-7 and HMGA2 [26].

In order to study the relationship and role of Mir-let-7 and HMGA2 in regulating the proliferation, migration, and invasion of colon cancer cells, we first detected the expression of miR-let-7 and HMGA2 in colon cancer cell line HCT116 by PCR and Western blot. It was found that the expression of miR-let-7 was downregulated and the expression of HMGA2 was upregulated in HCT116 cells. This indicates that miR-let-7 and HMGA2 are abnormally expressed in colon cancer. The detection of HMGA2 expression in HCT116 cells after transfection upregulated or inhibited miR-let-7 showed that miR-let-7 can negatively regulate the HMGA2 gene. In addition, MTT experiments proved that upregulation and inhibition of miR-let-7 can inhibit or promote the proliferation of colon cancer cell line HCT116, and wound healing experiments and Transwell chamber experiments proved that upregulation and inhibition of miR-let-7 can inhibit or promote the migration and invasion ability of colon cancer cell line HCT116. These results confirm that miR-let-7 can inhibit the proliferation, migration, and invasion of colon cancer cells by inhibiting the expression of the target gene HMGA2.

In summary, the abnormal expression of miR-let-7 is an important factor affecting the proliferation, migration, and invasion of HCT116 cells, and it can promote or inhibit the biological behavior of cancer cells by targeting the expression of HMGA2. The research results have important molecular significance for the diagnosis and treatment of colon cancer in the future and provide ideas for the development of new gene targets.

## Figures and Tables

**Figure 1:** Expression of miR-let-7 and HMGA2 in colon cancer cell HCT116. (a) qRT-PCR detected the intracellular miR-let-7 mRNA expression level. (b) qRT-PCR detected the intracellular HMGA2 mRNA expression level. (c) Western blot detected the intracellular HMGA2 protein expression level; compared with FHC, ^*∗*^*p* < 0.05.

**Figure 2:** The expression of miR-let-7 in colon cancer cell HCT116 after transfection. (a) qRT-PCR detected the miR-let-7 mRNA expression level after miR-let-7 was upregulated by cells. (b) qRT-PCR detected the miR-let-7 mRNA expression level after miR-let-7 was inhibited by cells; compared with mimic-NC and inhibitor-NC, ^*∗*^*P* < 0.05.

**Figure 3:** miR-let-7 has a targeting relationship with HMGA2. Bioinformatics website and dual-luciferase report detected the relationship between miR-let-7 and HMGA2; compared with mimic-NC and inhibitor-NC, ^*∗*^*p* < 0.05.

**Figure 4:** The regulatory effect of miR-let-7 on HMGA2. (a) qRT-PCR detected the HMGA2 mRNA expression level after miR-let-7 was upregulated by cells. (b) qRT-PCR detected the HMGA2 mRNA expression level after miR-let-7 was upregulated by cells. (c) qRT-PCR detected the HMGA2 protein expression level after miR-let-7 was upregulated by cells. (d) qRT-PCR detected the HMGA2 protein expression level after miR-let-7 was inhibited by cells; compared with mimic-NC and inhibitor-NC, ^*∗*^*p* < 0.05.

**Figure 5:** The effect of upregulation of miR-let-7 on the proliferation, migration, and invasion of colon cancer cell HCT116. (a) MTT detected the cell proliferation ability. (b) Wound healing test detected the cell migration ability. (c) Transwell test detected the cell invasion ability; compared with mimic-NC, ^*∗*^*p* < 0.05.

**Figure 6:** The effect of inhibiting miR-let-7 on the proliferation, migration, and invasion of colon cancer cell HCT116. (a) MTT detected the cell proliferation ability. (b) Wound healing test detected the cell migration ability. (c) Transwell test detected the cell invasion ability; compared with inhibitor-NC, ^*∗*^*p* < 0.05.

**Table 1:** Related primer sequences.

Primer sequence	Forward (5′-3′)	Reverse (5′-3′)
miR-let-7	UUCUCCGAACGUGUCACGUTT	ACGUGACACGUUCGGAGAATT
HMGA2	AAGAAAGCAGAAGCCACTG	TCAGTTTCCTCCTGAGCAG
U6	ATACAGAGAAAGTTAGCACGG	GGAATGCTTCAAAGAGTTGTG
GAPDH	ACAGCAACAGGGTGGTGGAC	TTTGAGGGTGCAGCGAACTT

## Data Availability

The data analyzed during the current study are available from the corresponding author upon request.
